# Consideration of the diameter of superficial temporal arteries related to filler injections in the temporal region

**DOI:** 10.1111/srt.13674

**Published:** 2024-04-01

**Authors:** Jung‐Hee Bae, Soo Hyun Park, Kyu‐Ho Yi

**Affiliations:** ^1^ Department of Dental Hygiene Namseoul University Cheonan South Korea; ^2^ Made‐Young Plastic Surgery Clinic Seoul South Korea; ^3^ Division in Anatomy and Developmental Biology Department of Oral Biology Human Identification Research Institute BK21 FOUR Project Yonsei University College of Dentistry Seoul South Korea; ^4^ Maylin Clinic (Apgujeong) Seoul South Korea

**Keywords:** hyaluronic acid, needle, skin vascular ultrasonography, superficial temporal artery, vascular complication

## Abstract

**Background:**

The concavity of the temple due to adipose tissue atrophy from aging accentuates the zygomatic arch and lateral orbital rim, leading to an aged appearance. The use of hyaluronic acid filler in the temporal region has gained popularity due to its procedural simplicity and consistent outcomes.

**Objective:**

To evaluate the safety of administering hyaluronic acid filler in the temporal region concerning the frontal branch of the superficial temporal artery, which is at risk of injury.

**Methods:**

Empirical observations were conducted on the internal diameter of the frontal branch of the superficial temporal artery, a critical anatomical site for potential injury.

**Results:**

A significant proportion of the artery segments exhibited an internal diameter below 1 mm. Given that the outer diameter of an 18‐gauge cannula is 1.27 mm, this method can be considered a relatively secure approach for enhancing the temporal region.

**Conclusion:**

The use of an 18‐gauge cannula for hyaluronic acid filler administration in the temporal region appears to be a safe and effective method, with the potential risk to the frontal branch of the superficial temporal artery being minimal.

## 1 INTRODUCTION

Hyaluronic acid (HA) filler injection in the temporal region is a popular procedure due to its relative ease and predictable outcomes of temple augmentation.^1^ Filler injections can increase the volume in the temporal area and create a smoother appearance,^2^ however, during temporal filler procedures, anatomical layers, vascular distribution, and variations in the area must be taken into consideration.

The most common complication of filler injections in the temporal region is vascular complications. These complications may result from the filler being injected into blood vessels or causing vascular compression, leading to adverse effects such as skin necrosis (Figure 1).^3^ To minimize vascular complications, clinicians should consider not only injection techniques but also anatomical data, including vascular distribution, pathways, and diameters.

**FIGURE 1:** Consequences arising from the vascular infiltration of the superficial temporal artery complication. This occurred on the 32nd day subsequent to the ischemic injury. Hyaluronidase, totaling 500 Units, was administered thrice, spaced at intervals of 8 h each.

## 2 ANATOMY OF THE TEMPORAL REGION

The temporal region is anatomically composed of several layers.^4^ Starting from the surface, it consists of the skin layer, subcutaneous layer, superficial temporal fascia, deep temporal fascia, temporalis muscle, and temporal bone. On the surface of the temporalis muscle, there are two layers of fascia. The superficial temporal fascia is a fascial layer located beneath the skin, surrounding blood vessels, and continuing with the SMAS (superficial musculoaponeurotic system). Beneath it, there is the deep temporal fascia, and inferiorly, the temporal muscle is located.

One of the significant blood vessels to consider in the temporal region is the superficial temporal artery. In the temporal area, the frontal branch and zygomatico‐orbital artery of the superficial temporal artery are noteworthy.^5^ Marano et al. reported anatomical data on the superficial temporal artery. The artery is surrounded by the superficial fascia and travels upward, passing through the temple area. Mostly, it divides into frontal and posterior branches near the temple area. Occasionally, there may be only one frontal branch or only a posterior branch. The diameter narrows as it moves away from the temple area. Approximately 3 cm above the temple area, before bifurcation, the diameter of the artery is around 1.9 mm. At a location approximately 3 cm above the zygomatic arch, the superficial temporal artery bifurcates. The thickness of this bifurcation point is reported to be 1.9 mm. Previous research has compared the thickness difference between the external and internal diameters of facial blood vessels, revealing that about 60% of the outer diameter is composed of the inner diameter.^6^ This implies that the internal diameter at the bifurcation point is approximately 1.2 mm, and at a distance of 7 cm from the bifurcation point, it reduces to about 0.6 mm. In other words, for the frontal branch of the superficial temporal artery on the temple side, which is the most vulnerable to damage, it is observed that most parts have an internal diameter less than 1 mm. Considering that the outer diameter of an 18‐gauge cannula is known to be 1.27 mm, it may be a relatively safe method for augmenting the temporal region (Figure 2).

**FIGURE 2:** The figure illustrates the techniques for injecting filler into the temple area using an 18‐gauge cannula. The yellow point indicates the new entry point for the filler injection, and the injection layer is chosen between the superficial and deep temporal fascia. The presence of the superficial temporal artery in the frontal and parietal regions has been observed.

## 3 CLINICAL APPROACHES IN TEMPORAL AUGMENTATION

The temporal region consists of multiple layers, all of which can be targeted for filler injections. One approach suggests injecting filler deep into the periosteal layer between the temporal bone and the temporalis muscle.^7^ This targets the layer just below the temporalis muscle and requires a significant amount of filler in a deeper plane than the muscle. However, in this approach, the filler may spread within the muscle and dissipate quickly due to shearing forces,^8^ leading to the formation of nodules that can be challenging to remove.

Another approach suggests injecting between the superficial temporal fascia and the deep temporal fascia.^9^ Lee et al. reported high patient satisfaction and observed no complications when injecting in the space between these fascial layers, leading to the conclusion that it is a safe area for temporal filler injections.^10^ Moreover, this approach allows for augmentation with relatively smaller amounts of filler. When using a cannula for injection, the superficial temporal fascia is more easily pierced, while the deep temporal fascia is more challenging to penetrate, making the injection between these fascial layers a more straightforward approach.

For the injection technique in the temporal region, the suggested injection point is 1 cm lateral and 1 cm superior to the lateral end of the eyebrow.^7^ This point is considered relatively safe from blood vessels compared to other areas in the temporal region. However, the reproducibility of this injection point might vary from individual to individual, as it is based on the reference of the eyebrow and hairline. Utilizing ultrasound guidance to confirm the absence of blood vessels during the injection can enhance the safety of the filler procedure.^10^, ^11^

## 4 CASE

A 30‐year‐old female patient with hollow areas on her temples underwent a procedure involving the injection of 3 cc of hyaluronic acid filler, with 1.5 cc administered to each side. The injection was performed approximately 1 cm above the frontotemporal region, a craniometric landmark, along the superior temporal fusion line.

For the filler injection, an 18‐gauge cannula was used, and the injection plane was targeted at the supraperiosteal layer, situated between the periosteal layer and the ROOF on the forehead. In the temple area, the cannula approached the supra‐deep temporal fascia layer, between the deep temporal layer and the subSMAS fat. During the injection, the cannula was carefully inserted, gently scratching the surface of each layer after reaching the periosteal layer and the deep temporal fascia layer of the temple. Due to the relatively firm and elastic nature of these two layers, the risk of cannula‐induced damage was minimal.^12^ Throughout the procedure, an ultrasound (US) imaging system (14‐MHz B‐mode operation, Sono‐Finder, N‐finders, Republic of Korea) was utilized to visualize the injection site structures and the cannula's position (Figure 3).

**FIGURE 3:** The figure demonstrates the procedure of ultrasonographic‐guided filler injection into the patient's temple. Linear reflective echoes can be seen deep to the needle (arrowheads), and certain structures such as RA (reverberation artifact), STL (superior temporal line), DTF (deep temporal fascia), S (superficial), and L (lateral) are identified. The observation has been conducted by Sono‐Finder (14‐MHz B‐mode operation, N‐Finders, Republic of Korea).

Both the clinicians and the patient expressed satisfaction with this novel injection method, and no side effects were reported following the procedure. A representative case of a patient who underwent this technique exhibited noticeable improvements in temple augmentation (Figure 4).

**FIGURE 4:** The figure displays a comparison of the augmentation achieved through filler injection in a 30‐year‐old female patient. The photographs show the patient before (A) and immediately after (B).

## 5 DISCUSSION

The aesthetic enhancement of the temples through filler injections has gained widespread popularity due to its procedural simplicity and reliable outcomes. However, these procedures present certain risks, especially when considering the anatomical intricacies and vascular complications in the temporal region.

Anatomical considerations play a pivotal role in determining the safety and efficacy of filler injections. The temporal region comprises distinct layers, including the skin, subcutaneous tissues, superficial and deep temporal fascia, temporalis muscle, and the temporal bone. The superficial temporal artery, particularly its frontal branch and zygomatico‐orbital artery, holds significance in this area.^13^ Studies, such as Marano et al. have highlighted the anatomy of the superficial temporal artery, emphasizing its vulnerability to damage during procedures due to its diminishing internal diameter, often below 1 mm, notably on the temple side. These observations are crucial, considering that the outer diameter of an 18‐gauge cannula frequently used in filler injections measures 1.27 mm. This insight suggests a relatively secure approach for augmenting the temporal region, given the disparity in cannula size and arterial diameter.

Clinical approaches for temporal augmentation involve injecting fillers into different layers of the temporal region. Techniques targeting the periosteal layer between the temporal bone and temporalis muscle or between the superficial and deep temporal fascia layers have been proposed. While injecting deep into the periosteal layer offers volume enhancement, it risks filler dispersion within the muscle, potentially leading to nodules. In contrast, injecting between the superficial and deep temporal fascia layers is deemed safer and effective, allowing augmentation with smaller filler quantities. Clinicians usually target a specific injection point, approximately 1 cm lateral and superior to the lateral eyebrow end, for temporal filler injections. This reference point, while relatively safer, might vary among individuals, emphasizing the importance of personalized techniques. Utilizing ultrasound guidance to confirm the absence of blood vessels during injection further enhances procedural safety.

A presented case illustrated a novel injection technique for temple augmentation, utilizing an 18‐gauge cannula targeting the supraperiosteal and supra‐deep temporal fascia layers. The use of ultrasound imaging during the procedure ensured accurate placement and minimized risks, resulting in both clinician and patient satisfaction with noticeable improvements in temple augmentation without any reported side effects.

In conclusion, this study underscores the importance of anatomical understanding in temporal filler procedures, emphasizing the vulnerability of the frontal branch of the superficial temporal artery in the temple area. Techniques targeting specific layers within the temporal region, alongside careful cannula size considerations and ultrasound‐guided injections, contribute significantly to safer and more effective temple augmentation. However, further research and larger‐scale studies are imperative to validate these findings and refine techniques for optimal outcomes in temporal filler procedures.

## AUTHOR CONTRIBUTIONS

All authors have reviewed and approved the article for submission. Conceptualization, Kyu‐Ho Yi Writing—Original Draft Preparation, Kyu‐Ho Yi, Jung‐Hee Bae Writing—Review & Editing, Kyu‐Ho Yi, Jung‐Hee Bae Visualization, Kyu‐Ho Yi, Jung‐Hee Bae, Soo Hyun Park Supervision, Kyu‐Ho Yi, Jung‐Hee Bae Consideration of the Diameter of Superficial Temporal Arteries Related to Filler Injections in the Temporal Region

## CONFLICT OF INTEREST STATEMENT

The authors have all considered the conflict of interest statement included in “Author Guidelines.” To the best of our knowledge, no aspect of the authors’ current personal or professional life might significantly affect the views presented on this manuscript. The authors declare no conflicts of interest.

## Data Availability

The data that support the findings of this study are available from the corresponding author upon reasonable request
